The article "miRNA-187-5p Regulates Osteoblastic Differentiation of Bone Marrow Mesenchymal Stem Cells in Mice by Targeting ICAM1" was retracted in 2024. Reasons: signs of a paper mill; compromised peer review; unreliable results or conclusions.

# miRNA-187-5p Regulates Osteoblastic Differentiation of Bone Marrow Mesenchymal Stem Cells in Mice by Targeting ICAM1

**DOI:** 10.1155/2020/6139469

**Published:** 2020-12-11

**Authors:** Yi Sun, Xin Wang, Guanghua Chen, Chengchao Song, Xinnan Ma, Yutuo Fu, Chao Feng, Jinglong Yan

**Affiliations:** ^1^Department of Orthopeadics, The 2nd Affiliated Hospital of Harbin Medical University, 148 Baojian Road, Harbin 150081, China; ^2^Physical Education and Research Office, Harbin Medical University, Harbin 150081, China; ^3^Department of Orthopedics, Heilongjiang Provincial Hospital, Harbin 150010, China; ^4^Department of Pharmacology, Harbin Medical University, Harbin 150081, China

## Abstract

Osteoporosis (OP) is a common bone metabolic disease, the process of which is fundamentally irreversible. Therefore, the investigation into osteoblastic differentiation of bone marrow mesenchymal stem cells (BMSCs) will provide more clues for OP treatment. In the present study, we found that microRNA-187-5p (miR-187-5p) played a key role on osteoblastic differentiation, which was significantly upregulated during osteogenic differentiation of BMSCs in mice. Moreover, overexpression of miR-187-5p suppressed osteoblastic differentiation of BMSCs through increasing alkaline phosphatase (ALP), matrix mineralization, and levels of Osterix (OSX), and osteopontin (OPN) as well as runt-related transcription factor 2 (Runx2) *in vitro*. The results *in vivo* indicated that the upregulation of miR-187-5p enhanced the efficacy of new bone formation in the heterotopic bone formation assay. Luciferase reporter assay and western blot analysis revealed that miR-187-5p was involved in osteogenesis by targeting intracellular adhesion molecule 1 (ICAM-1). Furthermore, ICAM-1 silence inhibited osteoblastic differentiation of BMSCs. Taken together, our results suggested for the first time that miR-187-5p may promote osteogenesis by targeting ICAM-1, and provided a possible therapeutic target for bone metabolic diseases.

## 1. Introduction

Millions of older adults throughout the world are suffering from osteoporosis, especially in postmenopausal women. Osteoporosis (OP) is the most common metabolic bone disease because of the unbalance between new bone formation by osteoblasts and old bone resorption by osteoclasts [1]. Osteoporosis is caused by the dysfunction of bone metabolism which is characterized with low bone mass, leading to reduced bone mineral density and subsequent elevated risk of fractures [2]. Bone marrow-derived mesenchymal stem cells (BMSCs) are stromal cells with the potential of continuous self-renewal and multidirectional differentiation to osteoblasts, chondrocytes, and adipocytes [3, 4]. It has been reported that reduced bone formation and increased marrow fat accumulation are major characterizations of age-related osteoporosis [5]. Thus, enhancing BMSC differentiation into osteoblasts may increase bone formation and improve the pathophysiological status of OP.

MicroRNAs (miRNAs) are a class of small molecule noncoding RNA that is highly conserved in diverse organisms. In the process of biological evolution, microRNA can identify the 3′-untranslated region (3′-UTR) of the target gene mRNA by its base pairing principle, degrading or inhibiting the transcription of target mRNA [6–8]. Additionally, miRNAs participate in multiple diseases, such as osteoarthritis [9], acute lymphoblastic leukemia [10], lung cancer [11], and cervical cancer [12, 13]. Recently, it has been found that dysfunction of miRNAs is considered a critical pathological factor in OP [14]. Growing evidence has shown that miRNAs play an important role in multidirectional differentiation potential of BMSCs [15, 16]. LRP3/hsa-miR-4739 axis in hBMSCs affects the balance between osteogenic and adipocytic differentiation [4]. In addition, miR-139-5p has an impact on BMSC osteogenesis most probably by directly targeting CTNNB1 and frizzled 4 (FZD4) through the Wnt/beta-catenin pathway [16].

miR-187-5p has been widely studied in recent years as a tumor suppressor in cervical cancer [12, 13], bone tumor [17], lung cancer [11, 18], and urologic neoplasms [19]. It has been investigated that miR-187 could suppress S100A4 expression through binding with S100A4 mRNA 3′-UTR in osteosarcoma cells [17]. In lung cancer, miR-187 contributes to the initiation of metastasis through regulating mitogen-activated protein kinase (MAPK) and phosphatidylinositol-3-kinase/protein kinase B (PI3K/PKB) pathways. Upregulation of miR-187 suppresses cervical cancer cell migration and invasion via directly targeting MAPK12. Besides, overexpression of miR-187-3p inhibits osteoblastic differentiation by reducing cannabinoid receptor type 2 (CNR2) expression [20]. However, no report has demonstrated the relationship between miR-187-5p and osteogenic differentiation. Therefore, we further tested whether the miR-187-5p expression changes during BMSC osteogenesis.

Intracellular adhesion molecule 1 (ICAM1) could regulate bone remodeling by promoting osteoclast formation and is considered critically important in various inflammatory bone diseases such as tuberculosis, inflammatory arthritis, or osteomyelitis. ICAM-1 is also known as CD54, which is a glycoprotein belonging to the immunoglobulin superfamily, the superfamily of proteins including antibodies and T-cell receptors. ICAM1 is lowly expressed on the surface of osteoprogenitor cells while is upregulated by proinflammatory cytokines including TNF-*α* and IL-*β* [21, 22]. However, whether ICAM-1 is associated with osteoporosis due to aseptic inflammation has not been reported. Here, the expression of miR-187-5p was measured during the osteogenic differentiation of BMSCs and the effects of miR-187-5p on alkaline phosphatase (ALP), matrix mineralization, Osterix (OSX), and osteopontin (OPN) as well as runt-related transcription factor 2 (Runx2) were also detected, which are key factors of osteogenesis. Furthermore, we found that ICAM-1 was a target of miR-187-5p and thus, the regulatory mechanism of miR-187-5p/ICAM-1 in BMSCs into osteogenic differentiation was evaluated, which could reveal a new mechanism and provide a novel therapeutic target for age-related bone loss.

## 2. Materials and Methods

### 2.1. Animals

The 6-week-old BALB/c-nu mice (18-20 g weight) were obtained from the Experimental Animal Center of the Second Affiliated Hospital of Harbin Medical University. Additionally, all animal protocols followed the Guide for the Care and Use of Laboratory Animals published by the US National Institutes of Health. All animal experimental procedures were performed strictly in accordance with the Ethics Committee of Harbin Medical University (No. sydwgzr2018-217).

### 2.2. Culture of BMSCs

Primary C3H10T1/2 BMSCs were purchased from Cyagen Biosciences Inc. Then, 1 × 10^5^ cells/cm^2^ BMSCs were seeded into 6-well plates and cultured with BMSC culture medium (Cyagen Biosciences, USA) supplemented with 100 U/mL penicillin-streptomycin, 10% fetal bovine serum (FBS), 10 nmol/L dexamethasone, 1% glutamine, 10 mmol/L *β*-glycerophosphate, 0.2 mmol/L l-ascorbic acid, and bone morphogenetic protein- (BMP-) 2 (Changzhou Kangfulai Medical, China). Next, the BMSCs were collected to eliminate the thrombus and seed into 25 cm^2^ flasks (Corning, USA) followed by incubating at 37°C in a humidified atmosphere with 95% air and 5% CO_2_ (Thermo, USA). After the cells were cultured to 80%~90% confluence, the culture medium was discarded, and 2 mL of BMSC osteoblastic differentiation medium containing 1% glutamine, 10% FBS, 1% penicillin-streptomycin, 1% b-glycerophosphate, 0.2% ascorbic acid, and 0.01% dexamethasone was added. The medium was replaced every 3 days. Finally, cells were detached with 0.25% trypsin (Cyagen Biosciences, USA) and collected for ARS staining, ALP staining, qRT-PCR, or western blot after being cultured with osteoblastic differentiation culture medium for 14 days. BMSCs between the third and fifth passages were used in this study. All cell experiments were repeated three times.

### 2.3. Cell Transfection

Liposome transfection was used, and the transfection reagent X-treme was used for cell transfection. Two hours before transfection, the medium in the clean orifice plate was discarded under aseptic conditions, and the opti-MEM-free medium was added to the hungry cells. At the time of transfection, the final concentration of miR-187-5p mimics and the negative control (NC) was 50 nM, and that of miR-187-5p inhibitor and NC was 100 nM. Fresh culture medium was replaced 6 h after transfection, and follow-up experiments were conducted 24 h later. Mmu-miR-187-5p mimic, mmu-miR-187-5p inhibitor, and NCs were synthesized by GenePharma (China). The sequences of mmu-miR-187-5p mimics were as follows: primary chain, 50-AGGCUACAACACAGGACCCGGG-30, and passenger chain, 50-CGGGUCCUGUGUUGUAGCCUUU-30. The sequence of mmu-miR-187-5p inhibitor was 50-CCCGGGUCCUGUGUUGUAGCCU-30.

### 2.4. Alkaline Phosphatase (ALP) Staining and Quantification

To detect matrix mineralization deposition by ALP staining, 2 × 10^4^ cells/cm^2^ BMSCs were seeded in 24-well plates and cultured for 14 days with osteogenic differentiation medium. In brief, BMSCs in 24-well plates were mildly rinsed with phosphate-buffered saline (PBS) (Solarbio, China) three times and then fixed by 95% ethanol (Tianjin Fuyu Fine Chemical, China) at room temperature (RT) for 15 minutes followed by washing with PBS three times. BMSCs were stained with the ALP neutral buffer staining solution (2% sodium pentobarbital, 3% *β*-glycerophosphate disodium salt hydrate, 2% calcium chloride, and 2% magnesium sulfate, pH 9.4) for 4~6 h at 37°C. Next, 2% cobalt nitrate (Tianjin Haijing Fine Chemical, China) was added to incubate cells for 10 minutes at RT. After washing cells with PBS three times, cells were incubated with 1% ammonium sulfide (Tianjin Fuyu Fine Chemical, China) for 2 minutes at RT and washed with PBS three times. Then, the stained cells were photographed by a standard Nikon light microscopy (ECLIPSE TS100). According to the instructions of ALP activity detection kit (Beyotime, Shanghai, China). 200 *μ*L termination solution was added to terminate the reaction. The absorbance was measured at 420 nmol/L. According to the definition of enzyme activity, the activity of alkaline phosphatase was calculated.

### 2.5. Alizarin Red S (ARS) Staining and Quantification

To further identify matrix mineralization deposition by ARS staining, 2 × 10^4^ cells/cm^2^ BMSCs were seeded in 24-well plates and cultured for 14 days with osteogenic differentiation medium. Next, BMSCs were mildly washed three times with distilled water and fixed with 4% paraformaldehyde (PFA) (Tianjin Fuyu Fine Chemical, China) for 10 minutes at RT. Then, cells were rinsed with distilled water three times and stained with 2% ARS staining solution (Cyagen Biosciences, USA) for 15 minutes at RT. Subsequently, stained cells were washed with distilled water and photographed by a standard Nikon light microscopy (ECLIPSE TS100, Nikon, Japan). For quantification of mineralization, the ARS released from the cell matrix into the cetylpyridinium chloride (Sigma-Aldrich, USA) was measured at 560 nm by a microplate reader (Tecan, Swizerland).

### 2.6. RNA Extraction and Real-Time qPCR

Total RNA was extracted by TRIzol reagent (Life Technologies, USA) from different groups of BMSC and measured by the NanoDrop 8000 (Pierce Thermo Scientific) to identify the concentration and purity. Next, cDNA was generated using the One-Step miRNA cDNA Synthesis Kit (HaiGene, China). Subsequently, qPCR was performed by a 7500 Real-Time PCR Detection System (Applied Biosystems, USA) using SYBR Green Master Mix (Roche Applied Science, Germany). The expression level of U6 gene served as reference. Steps of qPCR were as follows: 95°C for 5 minutes, 40 cycles of 95°C for 15 seconds, 60°C for 30 seconds, and 72°C for 30 seconds.

### 2.7. Western Blot Analysis

BMSCs were lysed using radioimmunoprecipitation assay (RIPA) buffer containing protease inhibitor cocktail (Roche Applied Science, Germany). Next, protein fractions were collected by centrifugation at 13500 × g at 4°C for 15 min, and supernatants were collected for the subsequent analysis. Equal amounts (15 mg) of protein from each sample subjected to 12.5% SDS-PAGE and wet-transferred to nitrocellulose (NC) membrane (Millipore, Billerica, USA). The NC membranes were blocked with 5% nonfat dry milk in Tris-buffered saline (TBS) for 60 min at RT and incubated with primary antibodies overnight at 4°C. Primary antibodies applied in this study were listed as follows: Osterix (1 : 1000, Abcam, USA), OPN (1 : 1000, Abcam, USA), Runx2 (1 : 1000, Abcam), ICAM-1 (1 : 1000, Abcam, USA), and tubulin (1 : 1000, Abcam, USA). After washing with TBS containing 0.1% Triton X-100 (TBST) three times, the NC membranes were incubated in secondary antibodies (horseradish peroxidase-conjugated, 1 : 2000, Cell Signaling Technology, USA) followed by rinsing repeated 4 times at RT. Finally, immunoreactive bands were detected by the Odyssey Infrared Imaging System.

### 2.8. Dual-Luciferase Reporter Analysis

According to the target gene prediction software TagetScan, mmu-miR-187-5p and its putative binding site on the 3′-UTR of ICAM-1 mRNA were predicted. It was predicted that 143~149 nt on the 3′-UTR of Icam1 mRNA was the binding site of miR-187-5p (ACAUCGG). The target point sequence (WT) in the ICAM-1 mRNA 3′-UTR region and the sequence (Mut) after site-specific mutation of the WT target site were synthesized artificially (ACAUCGG—TGTAGCC). The fragment of ICAM-1 mRNA 3′-UTR including the predicted binding site for miR-187-5p was amplified and subsequently cloned into the psi-CHECK2 vector. Moreover, mutations of the miR-187-5p binding site within the 3′-UTR of ICAM1 mRNA were generated and subcloned into the psi-CHECK2 vector (Promega, USA). Finally, the success of recombinant plasmid vector was confirmed by sequencing. 2 × 10^4^ BMSCs were seeded in 24-well plates and cotransfected with the indicated ICAM-1 3′-UTR luciferase reporter vectors along with the miR-187-5p mimics/inhibitor or mimics-NC/inhibitor-NC by the Lipofectamine 2000 transfection reagent (Invitrogen, USA). The cells were harvested after 48 h of transfection, and the Dual-Luciferase Assay System (Promega, USA) was utilized to measure the luciferase activity.

### 2.9. Heterotopic Bone Formation Assay *In Vivo*

The protocol of heterotopic bone formation *in vivo* is shown in Figure 1. BMSCs were transplanted into immunodeficient mice after treatments with miR-187-5p mimics and mimics-NC. 1 × 10^5^ BMSCs were transfected with miR-187-5p mimics and mimics-NC for 24 h. Hydroxyapatite (HA) powder (40 mg, Zimmer Scandinavia, USA) was diluted with 100 *μ*L of standard growth medium and transferred into 1 mL syringe. Next, cells were trypsinized with the cultured BMSCs, and 5 × 10^5^ cells (in 200 medium) were carefully transferred on the top of HA powder in 1 mL syringe and incubated at 37°C for 4 h in 5% CO_2_. Furthermore, transfected BMSCs loaded onto HA granules per group to produce four implants (four mice per group). Each sample was given the same dose of the mixture. Finally, BMSCs were implanted subcutaneously on the dorsal side of BALB/C homozygous nude mice. The transplanted nude mice were then placed in a special feeding room for 8 weeks. All the animal experiments were approved by the Animal Care and Use Ethics Committee of Harbin Medical University.

### 2.10. Hematoxylin and Eosin (H&E) Stain and Masson's Trichrome Stain

After 8 weeks, the BALB/c-nu mice were euthanized for histological examinations. The implants (*n* = 4) were taken out and fixed by 4% PFA for 3 days followed by decalcification for 12 days in 10% EDTA (pH 7.4). The specimens were dehydrated after decalcification and then embedded in paraffin. 5 mm sections (*n* = 6) were cut and stained with H&E or Masson's trichrome stain (Solarbio, China). The semiquantitative image analysis was performed by ImageJ (NIH Image, USA).

### 2.11. Microcomputer Tomography (Micro-CT)

Micro-CT imaging was used to evaluate bone volume and microstructure under a SCANC micro-CT-100 instrument (SCANCO Medical, Switzerland). The implants were fixed in 4% PFA for 24 h and washed by PBS three times. For new-bone quantitation, three-dimensional structure images and the trabecular bone parameters of heterotopic bone including trabecular number (Tb.N), trabecular bone volume per tissue volume (BV/TV), trabecular separation (Tb.Sp), and trabecular thickness (Tb.Th) were analyzed by the Scanco software.

### 2.12. Statistical Analysis

Data were analyzed using GraphPad Prism 5 software. All experimental data were showed as mean ± standard error of the mean (SEM). One-way ANOVA was used to determine statistical significance of different groups. ^∗^*p* < 0.05, ^∗∗^*p* < 0.01, and ^∗∗∗^*p* < 0.001 were considered to be statistically significant.

## 3. Results

### 3.1. The miR-187-5p Expression during Osteogenesis

First, we did experiments about the alteration of miR-187-5p expression during BMSC osteogenesis. After 24 h of transfection of miR-187-5p mimics, mimics-NC, miR-187-5p inhibitor, and inhibitor-NC, BMSCs were cultured to osteogenic-induced medium (OM-CTL) and normal growth medium culture (NM-CTL), and the mineral nodules were determined by ALP and ARS staining. The results showed that compared with NM-CTL, the mineralization proportion was significantly increased on the 14th day (Figures 1(a) and 1(b)), indicating that the BMSC osteogenic induction model was successfully established. According to the qRT-PCR results, the expression levels of miR-187-5p were upregulated with OM treatment at day 7 and reached the peak on the 14th day (Figure 1(c)). Furthermore, the instant transfection efficiency of miR-187-5p mimics and inhibitor was measured by qRT-PCR and found statistically significant (Figure 1(d)).

### 3.2. The Function of miR-187-5p in the Osteogenic Differentiation of BMSCs *In Vitro*

To further study the effect of miR-187-5p on the osteogenic differentiation of BMSC, overexpression or knockdown of miR-187-5p in BMSCs at the cellular level was performed. After 14 days of osteogenic differentiation, ALP and ARS staining for BMSCs was used to observe the effect of overexpressed miR-187-5p on BMSCs' osteogenic differentiation in comparison with the negative control (NC). ALP activity and proportion of mineralization by ARS were dramatically increased by miR-187-5p mimics (Figures 2(a) and 2(b)), which were reduced by miR-187-5p inhibitor at the meantime (Figures 3(a) and 3(b)) in comparison with NC mimics or the NC inhibitor group. The ARS and ALP staining indicated that miR-187-5p mimics promoted BMSC osteoblast differentiation, while miR-187-5p inhibitor prevented the differentiation, suggesting that overexpression of miR-187-5p could significantly increase the number and area of mineralized nodules in BMSCs, effectively promoting osteogenic differentiation of BMSCs. Similarly, western blot assays suggested that the protein levels of Osterix, Runx2, and OPN were upregulated in response to miR-187-5p mimics (Figures 2(c)–2(e)), while downregulated after miR-187-5p inhibition (Figures 3(c)–3(e)) in comparison with the mimics-NC or inhibitor-NC group. The above results indicated that overexpression of miR-187-5p could significantly promote osteogenic differentiation of BMSCs.

### 3.3. Effects of miR-187-5p Upregulation on Bone Formation *In Vivo*

To determine whether miR-187-5p expression stimulated bone-forming capacity *in vivo*, BMSCs were mixed with the osteoconductive carrier HAP and implanted subcutaneously in nude mice of heterotopic bone formation (Figure 4). Micro-CT may provide a direct and easy method for quantitation of formed bone *in vivo*, depending on parameters related to Tb.N, BV/TV, Tb.Sp, and Tb.Th. This animal model ensured that all implants were made with the same type of HAP granulate because the interpretation of the data assumed equal mean HAP particle size and distance between particles. Micro-CT showed that the ability of bone formation was obviously increased in BMSCs with miR-187-5p mimics, with bone volume-related analysis (Figure 5(a)). A significant increase in Tb.N, BV/TV, Tb.Sp, and Tb.Th in the miR-187-5p mimic group and mimics-NC group was observed by micro-CT, (Figure 5(a)). From the view of cross section of micro-CT, we also observed the increased bone formation in the miR-187-5p mimic group.

Furthermore, histological analysis of heterotropic bone in immunodeficient mice was performed in implants harvested after 8 weeks of subcutaneous transplantation of BMSC with HA. The paraffin sections were treated with H&E or Masson staining, and the results revealed that implantation of the miR-187-5p mimics led to an increase in the amount of heterotopic bone formed with miR-187-5p mimics compared to mimics-NC (Figure 5(b)). These results indicated that miR-187-5p upregulation enhanced bone regeneration.

### 3.4. ICAM-1 Is a Direct Target of miR-187-5p

Subsequently, to reveal the mechanism of miR-187-5p regulating the differentiation of BMSCs into osteoblasts, the potential target genes of miR-187-5p were explored through the online tools (TagetScan). ICAM-1 was a putative candidate gene of miR-187-5p because it had a potential miR-187-5p binding site in the 3′-UTR of its mRNA (Figure 6(a)). The luciferase fluorescence intensity of wild-type ICAM-1 was significantly reduced by miR-187-5p mimic, while miR-187-5p inhibitor had no effect on the luciferase fluorescence intensity of wild-type ICAM-1. In addition, both of miR-187-5p mimic and inhibitor could not regulate the luciferase fluorescence intensity of mutant ICAM-1. These results indicated that miR-187-5p bound to the ICAM-1 mRNA 3′-UTR region and regulated the expression activity of ICAM-1 (Figure 6(b)).

Furthermore, the results of western blot also confirmed that overexpression of miR-187-5p significantly reduced the protein expression of ICAM-1, while knockdown of miR-187-5p markedly increased ICAM-1 expression (Figure 6(c)).

### 3.5. The Role of ICAM-1 in BMSCs' Osteogenic Differentiation *In Vitro*

To further study the effect of ICAM-1 on BMSCs' osteogenic differentiation, knockdown of miR-187-5p by siRNA in BMSCs at the cellular level was performed. After 14 days of osteoblast induction culture, ALP and ARS staining in BMSCs was used to observe the effect of ICAM-1 silence on BMSCs' osteogenic differentiation compared with that of the NC group. ICAM-1 silence dramatically increased ALP activity and proportion of mineralization by ARS (Figures 7(a) and 7(b)). The ARS and ALP staining showed that ICAM-1 silence could significantly increase the number and area of mineralized nodules in BMSCs, effectively promoting osteogenic differentiation of BMSCs. Similarly, western blot assays suggested that the protein levels of Osterix, Runx2, and OPN were upregulated in response to ICAM-1 siRNA compared with those of the NC group (Figures 7(c)–7(e)). Consistent with the effect of miR-187-5p overexpression, ICAM-1 silence could significantly promote osteogenic differentiation of BMSCs.

## 4. Discussion

This study investigated the physiological function and mechanism of miR-187-5p by inducing the differentiation of mouse BMSCs *in vivo* and *in vitro*. We identified that miR-187-5p was a regulator of osteoblastic differentiation in BMSCs for the first time. Moreover, we demonstrated that miR-187-5p played a positive role on the differentiation of BMSCs into osteoblasts by directly targeting ICAM-1 mRNA. This study provided novel insights into the role of miRNAs on osteogenesis of BMSCs.

Osteoporosis is a systemic skeletal disease, which changes not only bone mass but also bone morphology, ultimately leading to the decline of bone mechanical properties [23]. Osteoporosis is a metabolic bone disease characterized by reduced bone mass, which can cause spinal deformity, bone pain, and osteoporotic fractures [24]. Currently, the treatment methods for osteoporosis mainly focus on increasing bone density, reducing further bone loss, supplementing vitamin D content, and promoting intestinal calcium absorption. Three types of drug therapy have been applied for osteoporosis, namely, bone resorption inhibitors, bone formation promoters, and bone mineralization promoters [23]. In addition to these existing treatments, it is extremely urgent to find effective new strategies to prevent the osteoporosis through improving bone formation.

BMSCs have the characteristics of self-replication and multidirectional differentiation potential and can be differentiated into a variety of connective tissue cells, such as adipocytes, osteoblasts, chondrocytes, and myoblasts [25, 26]. Studies for the osteogenesis of BMSCs may provide novel insights to the development of more effective manipulations for treatment of osteoporosis [27] and muscle injuries [26]. In the multidirectional differentiation potential of BMSCs, miRNAs play a role in regulating the differentiation of stem cells in different directions, and the miRNAs involved in regulating the multidirectional differentiation potential of different types of stem cells are also different [28–30]. For example, miR-19a-3p promotes the osteogenic differentiation of human-derived mesenchymal stem cells by targeting HDAC4 (PMID: 31248594). By contrast, miR-214 negatively regulates the osteogenic differentiation of BMSCs through downregulating BMP2 expression (PMID: 30703347). In addition, miR-488 suppresses psoralen-induced osteogenic differentiation of BMSCs by targeting Runx2 (PMID: 31485621). However, the role of miR-187-5p in the osteogenic differentiation of BMSCs remains unclear.

Previous studies have showed that miR-187-5p was related to non-small-cell lung cancer, acute lymphoblastic leukemia, and bladder cancer, but little is known about the role of miR-187-5p in the BMSCs [10, 18, 31]. Our data showed that overexpression of miR-187-5p significantly promoted the osteogenic differentiation of BMSCs.

Subsequently, the mechanism of miR-187-5p regulating BMSC osteogenic differentiation was studied. First, the target genes of miR-187-5p were predicted on the online TargetScan software, and intracellular adhesion molecule 1 (ICAM-1) was selected as the target gene of this study. The luciferase reporter assay confirmed that miR-187-5p could bind and target ICAM-1. Further studies showed that miR-187-5p played a positive role on osteogenic differentiation of BMSCs by targeting ICAM-1, which has been demonstrated to associate with osteogenic differentiation and bone regeneration [32]. It has been reported that ICAM-1 inhibits the osteogenesis of BMSCs, which is a new molecular target to accelerate bone regeneration and repair in the inflammatory microenvironment.

To verify that miR-187-5p promotes osteogenesis, we established an ectopic osteogenesis model in nude mice. Through H&E and Masson's trichrome stain, we found that after overexpression of miR-187-5p, osteoblasts significantly increased. Micro-CT may provide a direct and easy method for quantitation of formed bone *in vivo*. There was a significant increase in Tb.N and Tb.Th in the heterotopic ossification model. This data suggested that miR-187-5p also promoted BMSC osteogenesis *in vivo*. However, in our study, miR-187-5p transgenic mice were not utilized to explore the function of miR-187-5p in osteoporosis and further experimental studies are needed to determine whether miR-187-5p binds to other genes or participates in signal transduction during differentiation. These are limitations of the present study.

It was found that ICAM-1 significantly activates the p38/MAPK, ERK/MAPK, and JNK/SPAK pathways [33]. Importantly, blocking the ERK/MAPK pathway can save osteogenic differentiation. According to our previous study [34], we indicated that miR-92b-5p participates in the osteogenic differentiation of BMSCs by directly targeting ICAM-1. As new discoveries on the role of ICAM-1 are being reported, ICAM-1 could become a potential target for osteoporosis as well. Therefore, we believe that the mechanism of the action of mir-187-5p may be ultimately promote BMSC osteogenic differentiation by targeting the expression of ICAM-1.

In summary, we first confirmed that miR-187-5p not only promoted osteogenic differentiation of BMSC cells *in vivo* and *in vitro* but also effectively bound to the 3′-UTR region of ICAM-1 mRNA through base complementary pairing to regulate ICAM-1 expression in the posttranscriptional level. Thus, downregulating the expression of ICAM-1 protein by miR-187-5p could inhibit the osteogenic differentiation of mesenchymal stem cells.

## 5. Conclusions

In conclusion, our study confirmed the effect of miR-187-5p on BMSCs' osteogenic differentiation process and clarified its downstream target, thus providing a new drug target and new treatment strategy for osteoporosis.

## Figures and Tables

**Figure 1:** miR-187-5p was upregulated during osteogenic differentiation of BMSCs. (a) ALP staining was performed on day 14 after osteoblastic differentiation. Scale bar, 100 *μ*m. (b) ARS staining was performed on day 14 after osteoblastic differentiation. Scale bar, 100 *μ*m. (c) qRT-PCR analysis of the levels of miR-187-5p in BMSCs for 0 days, 7 days, and 14 days after osteogenic medium induction. (d) qRT-PCR was applied to detect transfection efficiency after transfection of miR-187-5p mimics, mimics-NC, miR-187-5p inhibitor, and inhibitor-NC for 24 h in BMSC cells. The data are presented as mean ± SEM of 3 independent experiments (*n* = 3). ^∗^*p* < 0.05 and ^∗∗∗^*p* < 0.001.

**Figure 2:** The overexpression of microRNA-187-5p promoted the osteogenic differentiation of BMSCs. (a) ALP staining was applied to detect the osteogenic differentiation of BMSCs. Scale bar, 100 *μ*m. (b) ARS staining was used to determine the osteogenic differentiation of BMSCs. Scale bar, 100 *μ*m. (c–e) The protein levels of OSX, OPN, and Runx2 in response to miR-187-5p expression, determined by western blot assays at 72 h after transfection. The data are presented as mean ± SEM of 3 independent experiments (*n* = 3). ^∗^*p* < 0.05, ^∗∗^*p* < 0.01, and ^∗∗∗^*p* < 0.001.

**Figure 3:** The knockdown of microRNA-187-5p inhibited the osteogenic differentiation of BMSCs. (a) ALP staining was used to determine the osteogenic differentiation of BMSCs. Scale bar, 100 *μ*m. (b) ARS staining was used to determine the osteogenic differentiation of BMSCs. Scale bar, 100 *μ*m. (c, d) The protein levels of OSX, OPN, and Runx2 in response to miR-187-5p inhibition, determined by western blot assays at 72 h after inhibition or NC transfection. The data are presented as mean ± SEM of 3 independent experiments. ^∗^*p* < 0.05, ^∗∗^*p* < 0.01, and ^∗∗∗^*p* < 0.001.

**Figure 4:** The protocol of heterotopic bone formation.

**Figure 5:** Effects of miR-187-5p upregulation on bone formation *in vivo*. (a) The ectopic bone formation of the graft was observed from the perspective of three different cross-sectional images by micro-CT scanning. Micro-CT analysis provides data on parameters related to BV/TV, Tb.N, Tb.Th, and Tb.Sp. (b) Histological analysis of heterotopic bone formation with H&E staining, Masson staining, and quantification of bone regeneration. The black arrows indicate the location of bone formation, while the red arrows indicate hydroxyapatite. Scale bar, 50 mm. ^∗∗^*p* < 0.01 and ^∗∗∗^*p* < 0.001. *n* = 3.

**Figure 6:** miR-187-5p regulated the expression of ICAM-1. (a) Putative binding sequence of miR-187-5p in the 3′-UTR of Icam1 mRNA. (b) Luciferase reporter assays was applied to testify the regulatory relationship between miR-187-5p and ICAM-1. (c) Western blot was applied to detect the effect of miR-187-5p overexpression or knockdown on ICAM-1 protein expression. ^∗∗^*p* < 0.01 and ^∗∗∗^*p* < 0.001, *n* = 3.

**Figure 7:** ICAM-1 silence promoted the osteogenic differentiation of BMSCs. (a) ALP staining was applied to detect the osteogenic differentiation of BMSCs. Scale bar, 100 *μ*m. (b) ARS staining was used to determine the osteogenic differentiation of BMSCs. Scale bar, 100 *μ*m. (c–e) The protein levels of OSX, OPN, and Runx2 in response to ICAM-1 silence, determined by western blot assays at 72 h after transfection. The data are presented as mean ± SEM of 3 independent experiments (*n* = 3). ^∗^*p* < 0.05, ^∗∗^*p* < 0.01, and ^∗∗∗^*p* < 0.001.

## Data Availability

Some or all data, models, or code generated or used during the study are available from the corresponding author by request.

## Abbreviations

ALP: Alkaline phosphatase
ARS: Alizarin red S
BMSCs: Bone marrow-derived mesenchymal stem cells
BV/TV: Bone volume per tissue volume
CNR2: Cannabinoid receptor type 2
FBS: Fetal bovine serum
FZD4: Frizzled 4
HA: Hydroxyapatite
HAP: Hydroxyapatite
H&E: Hematoxylin and eosin
ICAM-1: Intracellular adhesion molecule 1
MAPK: Mitogen-activated protein kinase
micro-CT: Microcomputed tomography
miRNAs: MicroRNAs
NC: Negative control
NC: Nitrocellulose
OD: Optical density
OP: Osteoporosis
OPN: Osteopontin
OSX: Osterix
PI3K/PKB: Phosphatidylinositol-3-kinase/protein kinase B
RIPA: Radioimmunoprecipitation assay
Runx2: Runt-related transcription factor 2
Tb. N: Trabecular number
Tb.Sp: Trabecular separation
Tb. Th: Trabecular thickness
UTR: Untranslated region.
